The article "Association of Insulin Resistance and Elevated Androgen Levels with Polycystic Ovarian Syndrome (PCOS): A Review of Literature" was published in 2022. Journal: J Healthc Eng.

# Association of Insulin Resistance and Elevated Androgen Levels with Polycystic Ovarian Syndrome (PCOS): A Review of Literature

**DOI:** 10.1155/2022/9240569

**Published:** 2022-03-21

**Authors:** Yalan Xu, Jie Qiao

**Affiliations:** ^1^Centre for Reproductive Medicine, Department of Obstetrics and Gynecology, Peking University Third Hospital, Beijing 100191, China; ^2^National Clinical Research Centre for Obstetrics and Gynecology, Beijing 100191, China; ^3^Key Laboratory of Assisted Reproduction (Peking University), Ministry of Education, Beijing 100191, China; ^4^Beijing Key Laboratory of Reproductive Endocrinology and Assisted Reproductive Technology, Beijing 100191, China; ^5^Research Units of Comprehensive Diagnosis and Treatment of Oocyte Maturation Arrest, Chinese Academy of Medical Sciences, Beijing, China

## Abstract

The polycystic ovary syndrome (PCOS) is the disease featured by elevated levels of androgens, ovulatory dysfunction, and morphological abnormalities. At reproductive stage of women, the rate of PCOS occurrence is measured as 6–10% and the prevalence rate may be double. There are different pathophysiological factors involved in PCOS, and they play a major role in various abnormalities in individual patient. It is clear that there is noteworthy elevation of androgen in PCOS, causing substantial misery and infertility problems. The overexposure of androgen is directly linked with insulin resistance and hyperinsulinaemia. It has been reported previously that PCOS is related to cardiac metabolic miseries and potently increases the risk of heart diseases. Endometrial cancer is also a serious concern which is reported with exceedingly high incidence in women with PCOS. However, the overexposure of androgen has direct and specific influence on the development of insulin resistance. Although many factors are involved, resistance to the insulin and enhanced level of androgen are considered the major causes of PCOS. In the present review, we have focused on the pathophysiology and major revolutions of insulin resistance and excessive levels of androgen in females with PCOS.

## 1. Introduction

The polycystic ovary syndrome (PCOS) is the disease featured by elevated levels of androgens, ovulatory dysfunction, and morphological abnormalities. According to NIH (National Institutes of Health), it can be defined as “hyperandrogenism with ovulatory dysfunction.” At reproductive stage of women, the rate of PCOS occurrence is measured as 6–10% and the prevalence rate may be double [1–4]. It is clear that there is noteworthy elevation of androgen in PCOS, causing substantial misery and infertility problems. Somehow, PCOS has also some environmental influences like obesity, as well as factors contributing to obesity. Most of the previous reports concluded that deformities associated steroidogenesis and follicular development are crucially involved in PCOS progression [4, 5]. PCOS generally exhibits constantly secreted levels of the gonadotropin-releasing hormone (GnRH), increased levels of the luteinizing hormone (LH), and insufficient follicle-stimulating hormone (FSH) secretion contributing to elevated secretions of the androgens and ovulatory dysfunction. Moreover, majority of the PCOS-suffering population develops insulin resistance, which in turn leads to the amplified secretion levels of the androgen, thereby decreasing the sex hormone-binding globulin secretions [6–11]. Genome research has been discovered numerous genes linked investigations such genes for the beta subunit of FSH, gonadotropin receptors, insulin receptor, neoplastic cells domain-containing protein 1A (DENND1A), differentially expressed in normal, and thyroid adenoma-associated protein (THADA). “Developmental programming” by environmental or hormonal influences may also add to the development of the PCOS. There are different pathophysiological factors involved in PCOS and they play a major role in various abnormalities in individual patient. It has been found that PCOS is related to cardiac metabolic miseries and potently increases the risk of heart diseases [11–16]. The mechanism of androgen biosynthesis in ovaries and adrenal gland is explained in Figure 1.

PCOS is found to be the major concern of women health and puts serious life-threatening conditions. Among the ratio of women suffering from PCOS, 50–80% are the obese women, 30–35% are those reported with impaired glucose tolerance, and 8–10% are found to be diabetic or having family diabetes history. The risk of PCOS is related to the history and severity of these influences [5, 16–20]. Generally, women with PCOS exhibit reduced levels of high-density lipoprotein (HDL) and amplified concentrations of triglycerides and low-density lipoproteins (LDL) cholesterols compared with normal women. LDL cholesterol differences appeared to play a significant role in PCOS, and it remains a major concern in most of women. However, sometimes LDL levels in normal range may lead to misconception as the activities of the LDL and HDL in PCOS women are sparse [21, 22]. The elevation of coronary artery calcium scores has been also described in PCOS women and high incidence is reported for the postmenopausal women with PCOS. Many reports provide evidence on the cardiovascular abnormalities in patients with history of PCOS. Endometrial cancer is also a serious concern which is reported with exceedingly high incidence in females with PCOS [21, 22]. The risk factors of the endometrial cancer in menopausal PCOS women include anovulation, heavy fats, and insulin resistance. The fear of chronic anovulation results in prolonged estrogen-mediated mitogenic activation of the endometrium with inadequate progesterone access to cause endometrial differentiation. Females with PCOS also face severe problems in pregnancy like risk of gestational diabetes mellitus, obstructive sleep apnea, and emotional distress [23–29]. Although many factors are involved, resistance to the insulin and high androgen are considered the major causes of PCOS. In the present review, we focus on the pathophysiology and major revolutions of insulin resistance and excessive levels of androgen in females with PCOS. The discussions are focused on insulin resistance, mechanism of insulin resistance, hyperandrogenism in PCOS, PCOS phenotypes, impacts of PCOS on physiological functions of the PCOS woman, and various treatments approaches for the treatment of PCOS, insulin resistance, and high secretions of androgens.

## 2. Insulin Resistance in PCOS

The actual understanding of insulin resistance can be explained by the requirement of excessive insulin for the metabolic activities, while, besides metabolic activities, insulin is also required for mitogenic and reproductive actions [24]. The rapid and fast glucose analysis make the researchers able to analyse insulin resistance. For this purpose, homeostatic model evaluation, quantitative insulin sensitivity check index, and fasting glucose and insulin levels have been established and utilized in clinical research and also metabolic investigations in PCOS [24–27].

In general, the obesity of abdomen in PCOS is the reason of insulin resistance possibly induced via subclinical swelling but whether the metabolically active intra-abdominal adipose tissues are augmented or not is unclear. However, it was previously investigated that the lower circulating adiponectin detection in PCOS justified subcutaneous adipose tissue as a dysfunctional adipose tissue compartment and having correlation with insulin resistance. Although different methods have been used for prevalence of insulin resistance, where it was found to be varied in PCOS women with respect to the detection method [28–31], more recent findings concluded that obesity is the main risk factor of insulin resistance in individuals suffering from PCOS. The investigations revealed that diagnostic criteria of insulin resistance have limited impact on the insulin resistance detection in PCOS women. Insulin resistance in PCOS patients is the main concern, and its prevalence and mechanism need to be investigated. In previous reports, it was found that large population of PCOS women is suffering from compromised glucose tolerance and type 2 diabetes mellitus (T2DM) [28, 29]. The statistically higher prevalence rate of the compromised glucose tolerance and T2DM serious threatening bell for healthy life. Few clinical studies have reported the glucose tolerance in PCOS women and T2DM risk in PCOS individuals. According to the findings of various studies, it was found that all those PCOS females who are obese and overweight are at greater risk of the disturbances in glucose metabolism and they required to check their glucose regularly with proper metabolic profiling [29–35].

## 3. Pathways of Insulin Resistivity in Patients with PCOS

Insulin is receptor binding hormone that binds to its membrane glycoprotein. This consists of two subunits *α* and *β*, associated with disulphide bonds. Subunit *α* is extracellular region responsible for the binding site, while subunit *β* is the intracellular region responsible for provoking intrinsic tyrosine kinase activity [36]. Ligand bindings lead to generating intrinsic tyrosine kinase activity in subunit *β* and initiate tyrosine phosphorylation. That further leads to the metabolic activities of insulin upon substrate binding, for example, glucose transport and glycogen synthesis [36, 37]. PCOS is a health issue for women and insulin resistance is one of the crucial issues that need to be emphasized. Insulin is an essential hormone for glucose metabolism and its sensitization is necessary for proper glucose uptake and metabolism [8, 38]. The cell surface receptor is homologous with the insulin-like growth factor 1 (IGF-1) receptor, so there is specific interaction for the binding of insulin to surface. The uptake of glucose is stimulated [19, 28, 39, 40]. The MAPK-ERK pathway initiation takes place, which initiates stimulation of a series of enzymes cascades. In previous studies on PCOS women, cellular and molecular mechanism of insulin was highlighted and glucose uptake in insulin target tissues like adipose and skeletal muscles was evaluated in both lean and obese women [20, 25]. When observed in PCOS patients, it was concluded that although the receptors affinities of insulin are similar in both PCOS women and normal females, decreased insulin binding was recorded at pancreatic *β*-cell in adipose tissues resulting in low glucose uptake and insulin sensitivity in PCOSs females compared to normal females. The fact might be due the reduced abundance of GLUT4 in subcutaneous adipose tissues in PCOS patients, which leads to insulin insensitivity [19, 20, 25, 28, 41, 42]. Besides the reduction in sensitivity of insulin, *β*-cell dysfunction is also one of the reasons for low disposition. However, still it is unclear whether the subunit *β* defected function is the primary cause of insulin resistance or it is secondarily involved in insulin resistance [43, 44]. To analyse insulin resistance in PCOS patients, proinsulin and insulin ratio can be a marker. In PCOS women, the ratio of proinsulin and insulin can explain the insulin resistance and activity of *β*-cell. It was found that, in obese and overweight PCOS patients, there was increased secretion of insulin followed by the excessive levels of proinsulin, which results in insulin resistance and hyperinsulinaemia [19, 20, 25, 28, 39, 40]. These studies explained the dysfunction of *β*-cell in PCOS women and insulin resistance mechanism. PCOS is a genetically contributed disorder in its pathogenesis and considered a hereditary condition. It has been shown that first relatives of PCOS history will have reproductive and metabolic issues and more investigations revealed that hyperinsulineaemia will be developed in the early stages of life and remain persistent throughout the puberty of girls with hereditary history of PCOS. In such cases, the subjects are at high risk for hyperinsulinaemia and insulin resistance, even if they are not diagnosed with PCOS. The follow-up study of peripubertal adolescent girls whose mothers were suffering from PCOS presented reduced disposition index persistently which proposes the dysfunction of pancreatic *β*-cell and this might be one of the genetic causes in first-degree relatives of the PCOS population. Another probable hereditary reason for insulin resistance in PCOS is a significant rate of SH2 domain-containing adaptor protein (Lnk) activity in PCOS female's ovarian cell lines, which suppresses the MAPK-ERK and phosphatidylinositol 3-kinase-AKT signaling responses to insulin. Previously, skin fibroblasts were for the intrinsic problems in in insulin function in PCOS because both hyperandrogenism and hyperinsulinaemia affect insulin sensitivity. When PCOS fibroblasts were assessed for insulin stimulated receptors autophosphorylation, there was reduced receptors stimulation as well as minimal insulin sensitivity. More importantly, immunopurification studies revealed that there was no mutation in receptor gene of insulin in PCOS patients [19, 36, 38, 40, 41].

## 4. Hyperandrogenism and PCOS

The genetically determined excessive secretions of androgens from ovary are the major concern in clinical evaluation of PCOS [45, 46]. The secretions of androgen at early stages are generally considered premature in PCOS and though to develop insulin resistance in prior stages. In visceral adipocytes, the disturbances in lipid metabolism result in insulin resistance. Nevertheless, the overexposure of androgen has direct and specific influence on onset of insulin resistance [47–52]. The increased secretion of androgen is associated with malfunctioning of islets of Langerhans, thereby compromising the pancreatic metabolic functions and causing hyperinsulinaemia. In preclinical studies, in PCOS women, it was found to be a major cause of T2DM. These facts revealed the direct relationship of overexposure of androgens with hyperinsulinaemia, insulin resistance, and T2DM in PCOS population [45–59]. The impact of insulin on hypersecretion of LH and androgen and its correlation with ovary, pituitary gland, and adrenal gland are illustrated in Figure 2.

Androgens belong to the family of steroid hormones and oversecretion of androgens is considered the main clinical manifesto of the PCOS. So, how androgens are biologically manufactured and regulated should be understood. Since androgens are very important for women's reproductive hormonal system, their normal synthesis and secretion are of prime importance. Androgens are critical female reproductive endocrine system hormones. Androgens include androstenedione (A4), dihydrotestosterone (DHT), dehydroepiandrosterone (DHEA), testosterone (T), and dehydroepiandrosterone sulfate (DHEAS). A4, DHEA, and DHEAS are regarded as precursors of T and DHT. Among these, only DHT and T have a direction with androgenic receptors. Androgens are majorly prepared ovaries and adrenal glands, while steroidogenic enzymes regulate their synthesis [60–64].

Besides this, in PCOS gonadotropin releasing was seen to have much more secretions of luteinizing hormone (LH) with normal abundance of the follicle-stimulating hormone (FSH). The increase in LH secretions in PCOS women may be due to pulsatile increase in the secretions of gonadotropin-releasing hormone (GnRH). Previous analysis raises the point that the change in GRH secretion might be due to defects in hypothalamus in PCOS populations. However, these complications are not only concerned with PCOS, but such changes have been also observed with hyperandrogenism in other cases like ovarian cancer, where there are increased secretions of androgens. The discussion based on previous literature declares that GRH releasing behaviour in correlation with hyperandrogenism in PCOS may be the secondary issue not involved primarily [65, 66]. Women suffering from PCOS generally exhibit hyperandrogenism with increased ovarian androgen as illustrated in Figure 3. The theca cells are the cells of ovary which are responsible for the production of androgens; these cells secrete amplified levels of androgen (androstenedione) and 17-hydroxyprogesterone. 17-Hydroxyprogesterone is a steroidal intermediate for the biosynthesis steps of androgens and glucocorticoids to retort the LH. The questions arise that such abnormalities originate from the theca cells from the ovary of PCOS patients and chronic anovulation-PCOS or from theca cells of the normal ovaries [67–69]. Insulin can have mimicking influences on the LH in women with PCOS. When theca cells from women with PCOS were passaged in tissue culture, they demonstrated elevated activity of numerous steroidogenic enzymes: 3-hydroxysteroid dehydrogenase, 17-hydroxylase/17-20 lyase, and 17-hydroxysteroid hydrogenase. The previously published reports revealed the fact that the amplification of the steroidogenic activity is intrinsic and presumably genetic and leads to blemishes in PCOS. The PCOS might be a morphological associate of these steroidogenic abnormalities [56–62, 70].

## 5. PCOS Phenotypes

There are 4 various phenotypes of the PCOS identified up till now which are as follows: Type A: polycystic ovaries [PCO], chronic anovulation [CA], and Hyperandrogenism [H]; Type B: chronic anovulation [CA] and hyperandrogenism [H]; Type C: polycystic ovaries [PCO] and hyperandrogenism [H]; and Type D: polycystic ovaries [PCO] and chronic anovulation [CA] [70, 71]. The type of PCOS is related to metabolism and cardiovascular health, as it has been observed that most of the PCOS women are obese with severe or mild metabolic deformities [19, 70, 71] and often face problems of dyslipidaemia, hyperinsulinaemia, insulin resistance, and other metabolic disorders [20]. The major discussion is on fabricating how PCOS phenotypes can be related to aging. Patients with phenotype A are investigated to have high insulin resistance and overexposure of androgens as compared to phenotype B. Phenotype D is generally characterized by the insulin resistance in obese condition even if there is no overexposure of androgens. Meanwhile, in case of type C, the scenario is different where cardiovascular risk is high which may be due to lack of insulin resistance in PCOS. Dyslipidaemia is a serious metabolic issue in PCOS correlated with the HDL and LDL cholesterol levels. According to a research on the PCOS population, both lean and obese PCOS women exhibit aberrant phosphatidylcholine and polyunsaturated fatty acids (PUFAs) levels as well as free fatty acids [71–73].

## 6. Impact of PCOS on Physiologic Functions

PCOS is a heterogeneous disease of endocrine system which is followed by various clinical and physiological abnormalities. It exerts harmful and pervasive effects on physiological as well as metabolic system, and these characteristics categorise PCOS as a disorder associated with metabolism. Various dysfunctions like insulin resistance, hyperinsulinaemia, obesity, dyslipidaemia, hypertension, elevating risk of developing T2DM, endometrial hyperplasia, and coronary artery diseases. Here, we discussed the impact of the PCOS on various physiological functions of the body.

### 6.1. Liver Function

The excessive aggregation of fats in liver is called nonalcoholic fatty liver disease (NAFLD) and presents high risk of T2DM and CVS in PCOS. NAFLD is characterized by the presentation of insulin resistance and obesity. These issues are specifically related to abnormalities in liver metabolism. In PCOS population, there is always a high risk of NAFLD because PCOS women usually have insulin resistance with metabolic dysfunctions and unconditional obesity. So, PCOS consequences are found to be associated with NAFLD [74, 75].

### 6.2. Cardiac Functions

It was concluded that all the PCOS phenotypes have serious cardiovascular risks in PCOS patients. Phenotypes, insulin resistance, hyperinsulinaemia, overexposure of androgens, and ovaries function are reported to display increased cardiovascular health risk for PCOS women [76–78]. The insulin resistance is associated with the inactivation of NO after release from endothelial cells and decreased production of nitric oxide (NO) and synthesis of vasoconstricting agents in excessive amounts; all these defects lead to impaired vasodilatation and cardiac muscles stiffness [79, 80]. Insulin resistance and hyperinsulinaemia also display hypertrophic effect directly and proceed with the endothelial dysfunction. Clinical reports revealed increased risk of cardiac dysfunctions in PCOS population [77–81].

### 6.3. Reproductive Functions

PCOS is a primary disorder of the ovaries and will directly affect the reproductive system and functions. The excessive secretions of insulin have been observed to cause amplified levels of estrogens and progesterone secretions in women with PCOS. Insulin receptors are responsible for mediating these effects. It was reported that the insulin activity in in vitro granulosa cells can be treated with troglitazone, where IGF-1 mitogenic pathways are increased with the therapy. Besides this, there was an amplification in the IGF-1 receptor in the follicle cells of PCOS patient. This occurred in all stages of development in PCOS women [82]. In the recently reported data, it was concluded that the activity of cortisol is defective in follicular fluid and granulosa cells in PCOS population, where insulin resistance can further lead to tissue-specific insulin resistance. Endometrium cancer is a health-depriving deadly disorder and PCOS women are at high risk to develop endometrium cancer because of the high incidence of insulin resistance and hyperinsulinaemia together with overexposure of androgens. In PCOS, there is always increased upregulation of insulin receptors that have the direct implication of insulin signaling, thereby leading to cardiogenesis and development of endometrium cancer [83]. It might be due to metabolic defects, proteins expression in endometrium with insulin activity, and faulty glucose metabolism. Furthermore, the insulin receptor expression and IGF-1 signaling synergistically contribute to the development of endometrium cancer in PCOS population. So, PCOS is one of the major reasons for establishing endometrium cancer [82–84]. In Figure 4, the mechanism of PCOS associated infertility is illustrated, which displays the reproductive defects in PCOS women. The PCOS leads to increased production of androgens and decreased sensitivity of the follicle-stimulating hormone receptors (FSHR) as illustrated in Figure 4. The increased production of the androgens leads to failure in dominant follicles development and corpus luteum. It is responsible for decreased production of aromatase and progesterone. On the other hand, decreased sensitivity of the FSHR also leads to decreased aromatase production that further decreases the production of estrogens. So, overall, the syndrome leads to decreased production of the estrogens and progesterone followed by infertility.

### 6.4. PCOS and Hypertension

Hypertension is a persistently elevated blood pressure that affects a large human population and leads to serious health issues [84]. In PCOS population, the existence of systemic arterial hypertension (SAH) is more usual and has high incidence. A survey conducted on SAH in PCOS women demonstrated that there are 40% more chances of SAH occurrence in PCOS women than in the normal women. SAH has specific and central contribution in the development of PCOS and secondary cardiovascular disorders [84–88]. According to clinical investigational studies, there is a major and specific relationship between hypertension and endocrine system, so any abnormality in endocrine system will be definitely associated with the hypertension. In PCOS, the defective endocrine system is commonly observed leading to hypertension [85]. Besides this, insulin resistance and metabolic defects have also more commonly occurring issues in PCOS women, resulting in increased incidence of hypertension [84, 85]. The insulin resistance results in hyperinsulinaemia and increased production of LH, consequently increasing the androgen secretions causing persistently high blood pressure in PCOS women [89, 90]. The critical clinical studies show that there is a high occurrence of hypertension in females with PCOS. Moreover, it should be clearly understood that women suffering from PCOS should always monitor their blood pressure regularly in order to avoid delayed management [89–91].

### 6.5. Inflammation in PCOS

PCOS also promotes basis for chronic low-grade inflammation and inflammation pathways including interleukin-6 (IL-6), TNF-a, and type 2 TNF receptors. The circulating C-reactive protein (CRP) observation also leads to the point that PCOS is concerned with low-grade chronic inflammation [81, 91]. The basis can also be displayed from excessive adipose tissues which is direct producer of the CRP [92, 93]. Additionally, CRP has a physiological purpose by increasing lipid absorption into foamy macrophages inside atherosclerotic plaques. CRP is a direct and specific biomarker of abnormally low inflammation, according to a study [94, 95]. In general, PCOS patients have mild risk of chronic inflammation but it is not reflective at molecular levels.

## 7. Treatment Options for Hyperandrogenism, Insulin Resistance, and PCOS

### 7.1. Exercise and Weight Loss

Exercise is the best treatment modality for all the embolic manifestations and is recognized as necessary as food for human health. In PCOS, exercise and weight losing activities have supreme importance because they will help in lowering the adipose tissues having a major contribution to insulin resistance and androgenism [89, 96, 97]. The fats deposits are the key factors for insulin resistance, hyperinsulinaemia, hyperglycemia, T2DM, and oversecretion of androgen, so losing fats, specifically abdomen fats, has a direct and positive impact on all the major issues in PCOS women. It is also investigated that exercise not only diminishes fats but also promotes the normal endocrine and adrenal functions [97]. Physical exercises and weight losing activities can result in complete recovery from the clinical characteristics of PCOS.

### 7.2. Pharmacological Mediation

Drug therapy is always considered prime requirement for PCOS, where drugs like pioglitazone, inositol, and metformin isoforms have been recognized as therapeutic regimens for reproductive abnormalities and metabolic disorders in PCOS. Metformin is an insulin-sensitizing hormone that is used in PCOS even without diabetes and exerts actions on adipose tissue, skeletal muscles, ovary, and endothelium, impacted by insulin resistance. Prolonged use of metformin in PCOS treatment can augment ovulation rate, regulate menstrual cycle, and decrease the androgens secretions [87, 98–100]. The combinatorial regimen of clomiphene and metformin is considered more beneficial than single therapy of clomiphene or metformin for ovulation and pregnancy in PCOS women [101]. Metformin had no impact on fasting glucose, serum lipids, or anthropometric characteristics in women with PCOS, although it may postpone the advancement of glucose intolerance. Other insulin-sensitizing agents have also been shown to be effective in the treatment of PCOS [102]. Pioglitazone and rosiglitazone are also considered effective in eliminating insulin resistance, abnormal glucose tolerance, hyperandrogenaemia, ovulation rate, and menstrual regularity in PCOS patients. The combination of metformin and pioglitazone is also reported to have synergistic clinical profile in PCOS women's treatment; however, it should be avoided if pregnancy is desired due to teratogenic effects [103]. Inositol is another novel insulin-sensitizing agent that withholds superb insulin-sensitizing efficiency in PCOS women. Insulin resistance is troublesome along with hyperinsulinaemia for PCOS population and needs further research for the radical treatments. Hypersecretion of androgen in PCOS is considered fatal and hereditary. Therefore, there is an unmet need to evaluate the pathogenic and molecular network of this syndrome, insulin resistance, and excessive secretion of androgen [102, 103]. The metabolic irregularities and malfunctioning lead to complications like obesity, excessive lipids aggregations, impaired glucose tolerance, hypertension, endometrium cancer, and hyperinsulinaemia [104, 105]. There is intended need for randomised clinical control trials for effective therapeutic approach in order to treat PCOS and its related complications.

### 7.3. Assisted Reproductive Technology (ART)

Women infertility is also a major concern in PCOS, where assisted reproductive technology (ART) is employed for the fertility purposes. In ART, ovary is hyperstimulated in order to regulate the growth of multiple follicles, but it is ineffective in most cases due to augmented response to gonadotropins [106, 107]. In vitro maturation (IVM) methods have been employed for the fertilization of women with PCOS. IVF and IVM-IVF methods are also used for the embryo implantation to PCOS women [106–108]. However, further clinical research is aimed at yielding specified model for the success of ART in PCOS women to get fertilized.

### 7.4. Laparoscopic Ovarian Drilling (LOD)

In 1984, laparoscopic ovarian drilling (LOD) was established to replace the invasive ovarian wedge resection surgery [109]. Currently, this technique is highly recommended and is developing pregnancy in 84% of the PCOS women who are facing infertility problems. LOD also augments insulin resistance and androgen production from ovaries. The improvements achieved with LOD have been observed to remain for a long time in 54% of the PCOS population. LOD is also a beneficial approach, as it results in low incidence of miscarriages in PCOS patients. LOD is also thought to be the first-line treatment when the CC treatment fails [26, 110–116]. These findings should be further evaluated for the confined use of LOD and its clinical benefits.

### 7.5. Oral Contraceptive Pills (OCPs)

Oral contraceptives pills (OCPs) are regarded first-line therapy for people with PCOS who are not pursuing pregnancy. Not only are OCPs helpful in regulating the menstrual cycle, but also they reduce the secretion of androgens and regulate other physical activities [117]. OCPs have been reported which can significantly decrease the risk of endometrium cancer. OCPs are a combination of estrogen and progestogen, where estrogen is intended to decrease the levels of LH and FSH; the reduction in LH and FSH levels leads to suppression of T secretions and reduces the secretion of androgens. Progestogen is generally recommended for low androgenic activity in women with PCOS [118, 119]. Three commonly used progestogens are desogestrel, cyproterone acetate, and drospirenone. As discussed earlier in this review, the PCOS population has high risk to develop disorders like insulin resistance, T2DM, hyperglycemia, abnormal glucose tolerance, enhanced levels of HDL and LDL cholesterols, hyperinsulinaemia, and so forth. Investigations in clinics revealed that OCPs can cause serious cardiac disorders like thrombosis, hypertension, insulin resistance, and myocardial infarction. These anomalies are thought to be having high risk in PCOS women compared to normal women and those who are on OCPs therapy. However, up till now, no clinical examination has been reported, to the best of our knowledge, regarding the metabolic effects of OCPs in PCOS population [118–122]. So, there is a great demand of clinical research in this area of interest because OCPs are the first-line treatment modality in females with PCOS. The recent interventions declared a new regimen with OCPs by adding metformin along with OCP, and the results found were satisfactory in reducing insulin resistance as well as decreasing the androgen production in PCOS population.

### 7.6. Dietary Therapy

Dietary therapy to reduce the weight of women with PCOS has a significant impact on metabolic conditions and is recognized to improve many PCOS issues like regulating androgen secretions, reducing insulin resistance, regularity of endocrine secretions, and menstrual cycle regulation [123, 124]. Weight loss can surely meet the goals of obtaining improved symptoms of PCOS and metabolic issues can intently resolve without medications. Moreover, the reproductive consequences in PCOS women can be improved with weight loss for those PCOS women who are interested in getting pregnant [123]. The weight loss results in high rates of pregnancy as well as decrease of the chances of miscarriages, suggesting weight loss significance for PCOS population. Dietary plan for weight loss is important and should be considered as first clinical regimen in order to live a healthy life with PCOS [125–128]. There is a need for clinical research and trials on the significance and effectiveness of dietary therapy for PCOS women.

## 8. Conclusion

Polycystic ovarian syndrome (PCOS) is considered as a major health issue. Women with PCOS face insulin resistance and overexposure of androgen, leading to a number of metabolic and reproductive abnormalities. These are considered the major causes of PCOS and other PCOS related manifestations. Herein, we have discussed the mechanism and treatment modalities of PCOS based on hypersecretion of androgen and insulin resistance. The current study gives concise and comprehensive outlook for the understanding of insulin resistance and androgen overexposure. We for the first time reported detailed review on the mechanism, pathophysiology, and treatment interventions for the insulin resistance and hypersecretion of insulin. The current study provides better understanding of the PCOS and provides a base for further exploration.

## Figures and Tables

**Figure 1:** Production of androgen in ovaries and adrenal gland. Biosynthesis of the androgens associated with the ovary and the adrenal gland.

**Figure 2:** Impact of insulin on hypersecretion of LH and androgen.

**Figure 3:** The basic mechanism of androgen overexposure in PCOS women [69]. The figure is cited with permission granted.

**Figure 4:** Schematic representation of PCOS associated infertility. The increased production of the androgens leads to failure in dominant follicles development and corpus luteum that is responsible for decreased production of aromatase and progesterone. Decreased sensitivity of the FSHR also leads to decreased aromatase production that further decreases the production of estrogens. So, overall the syndrome leads to decreased production of the estrogens and progesterone leading to infertility. H: anti-Mullerian hormone; PKA: protein kinase A; AC: adenylate cyclase; cAMP-response element binding protein:CREB.

## Data Availability

All the data can be requested from the corresponding author.
